The article "GAPLINC is a predictor of poor prognosis and regulates cell migration and invasion in osteosarcoma" was published in 2018. Journal: Biosci Rep.

# GAPLINC is a predictor of poor prognosis and regulates cell migration and invasion in osteosarcoma

**DOI:** 10.1042/BSR20181171

**Published:** 2018-10-10

**Authors:** Shian Liao, Sijia Zhou, Chao Wang

**Affiliations:** 1 Department of Bone and Soft Tissue Surgery, Affiliated Tumor Hospital of Guangxi Medical University, Nanning 530021, Guangxi, China; 2 Department of Orthopedics, First Central Clinical College, Tianjin Medical University, Nankai District 300110, Tianjin, China; 3 Department of Orthopedics, The First Affiliated Hospital of Kunming Medical University, Kunming 650032, Yunnan, China

**Keywords:** biomarker, GAPLINC, large intervening non-coding RNA, osteosarcoma

## Abstract

Gastric adenocarcinoma predictive long intergenic non-coding (GAPLINC) is a novel long non-coding RNA (lncRNA) and has been found to function as an oncogenic lncRNA in gastric cancer, colorectal cancer, and bladder cancer. The expression status and biological function of GAPLINC in osteosarcoma are still unknown. Thus, we analyzed the association between GAPLINC expression and clinicopathological characteristics in osteosarcoma clinical samples, and conducted loss-of-function study in osteosarcoma cell lines. In our results, GAPLINC expression is elevated in osteosarcoma tissues and cell lines, and correlated with advanced Enneking stage, present distant metastasis, and poor histological grade. Survival analyses indicated that GAPLINC expression was negatively associated with overall survival, and GAPLINC high-expression was an independent risk factor in osteosarcoma patients. The *in vitro* studies showed knockdown of GAPLINC depressed osteosarcoma cell migration and invasion via inhibiting CD44 expression, but no effect on cell proliferation. In conclusion, GAPLINC may serve as a potential biomarker for predicting prognosis and developing therapy for osteosarcoma.

## Introduction

Osteosarcoma is the most commonly malignant bone cancer and often occurs in children and adolescents with an incidence of 4.4 per million people worldwide [1,2]. Osteosarcoma is derived from primitive transformed cells, and characterized by locally aggressive growth and high metastatic potential [3]. Despite of advances in multidisciplinary treatment including surgery, chemotherapy, radiotherapy, molecular targeting therapy, and immunotherapy, the prognosis of osteosarcoma is still unsatisfactory [4–6]. According to epidemiological reports, the 5-year survival rate is approximately 70% for in-patients without metastatic diseases, and is no more than 30% for osteosarcoma patients with recurrent or metastasis [7,8]. Therefore, it is useful to elucidate the molecular basis of osteosarcoma progression for developing effective therapeutic agents and improving osteosarcoma patient’s prognosis

More and more evidence now shows that long non-coding RNAs (lncRNAs) serve as key roles in various biological processes including carcinogenesis [9–11]. Gastric adenocarcinoma predictive long intergenic non-coding (GAPLINC), a novel long intergenic non-coding RNA, is located in the human chromosome 18p11.31 with 924-bp transcript. Initially, GAPLINC was found overexpressed in gastric cancer tissues and to serve as a poor prognostic factor in gastric cancer patients [12]. Meanwhile, GAPLINC regulated tumor cell proliferation and migration through competing with CD44 for miR-211-3p [12]. Subsequently, the clinical significance and biological function of GAPLINC was also explored in colorectal [13–15] and bladder cancers [16]. However, the role of GAPLINC in osteosarcoma is still unknown. Therefore, the purpose of our study is to assess the clinical value of GAPLINC in osteosarcoma patients, and estimate the effect of GAPLINC on osteosarcoma cell proliferation, migration, and invasion.

The article "GAPLINC is a predictor of poor prognosis and regulates cell migration and invasion in osteosarcoma" was published in 2018. Journal: Biosci Rep.

## Materials and methods

### Clinical tissue specimens

One hundred and twenty-six osteosarcoma tissues and forty adjacent non-cancerous normal tissues were collected from osteosarcoma patients who underwent surgery at Affiliated Tumor Hospital of Guangxi Medical University, Affiliated Hospital of Tianjin Medical University, and The First Affiliated Hospital of Kunming Medical University. The pathologic diagnosis of all cases was confirmed by two pathologists. None of the patients had received chemotherapy or radiochemotherapy before pathologic diagnosis. Clinical tissue samples were snap-frozen in liquid nitrogen and stored at −80°C for the following study. Clinical data including the patient’s age, gender, Enneking stage, tumor size, distant metastasis, and tumor site were collected with uniform form. Informed consent was obtained from all patients, and the research method was approved by the Ethics Committee of Affiliated Tumor Hospital of Guangxi Medical University, Affiliated Hospital of Tianjin Medical University, and The First Affiliated Hospital of Kunming Medical University, and complied with the Declaration of Helsinki.

### RNA isolation and RT-qPCR

Total RNA was extracted from clinical specimens or cells with the TRIzol reagent (Invitrogen, U.S.A.) and transcribed into cDNA using superscriptase II (Invitrogen, U.S.A.) according to the manufacturer’s instructions. The cDNA was subjected to real time-polymerase chain reaction using Power SYBR^®^ Green PCR Master Mix (Invitrogen, U.S.A.). The following primers were used: GAPLINC: 5′-TGGACTCAGGCACGTTTACAG-3′ (forward) and 5′-TCATTGTTCTGGCCTCTGTCC-3′ (reverse); GAPDH: 5′-TGCACCACCAACTGCTTAGC-3′ (forward) and 5′-GGCATGCACTGTGGTCATGAG-3′ (reverse). GAPDH was utilized as an internal control.

The article "GAPLINC is a predictor of poor prognosis and regulates cell migration and invasion in osteosarcoma" was published in 2018. Journal: Biosci Rep.

### Cell culture and cell transfection

Osteosarcoma cell lines MG-63, HOS, SJSA-1, Saos-2, and the human normal osteoblast cell line hFOB1.19 were obtained from American Type Culture Collection. These cells were maintained in RPMI 1640 supplemented with 10% FBS, 100 U/ml penicillin, and 100 μg/ml streptomycin at 37°C with 5% CO_2_.

The siRNAs (siRNA-NC and siRNA-GAPLINC) were obtained from GenePharma Co., Ltd. For cell transfection, osteosarcoma cells were seeded in six-well plates at 5 × 10^5^ per well and transfected with siRNA by lipofectamine 3000 transfection reagent (Invitrogen, U.S.A.) referring to the manufacturer’s instructions. The transfection efficiency was verified by qRT-PCR at 48 h after transfection.

### Cell Counting Kit-8 assay

Osteosarcoma cells were transfected with siRNA-GAPLINC or siRNA-NC. Twenty-four hours after transfection, cells were transferred into 96-well plates at 2000 per well with six replicate wells. Cell viability was assessed day 1, 3, and 5. The absorbance at 450 nm was measured after incubation with 10 μl of Cell Counting Kit-8 (CCK-8) reagent (Dojindo, Japan) for 4 h.

### Cell migration and invasion assays

The 8-μm polycarbonate nucleopore filters (Corning Costar, U.S.A.) were used in cell migration and invasion assays. For migration analysis, osteosarcoma cells (1 × 10^5^ cells) were seeded in the upper chamber of a 24-well Transwell unit. The upper chamber contained serum-free medium and the lower compartment contained medium with 10% FBS. After 24-h incubation, the cells adhering to the lower surface of the filter were fixed and stained with crystal violet (Beyotime, China). The staining cells were counted in five representative fields.

For the invasion assay, the Transwell membranes were precoated with Matrigel (BD Biosciences, U.S.A.) at 37°C for at least 4 h to form a reconstructed basement membrane. The procedure was the same with migration assay.

### Western blot

Total proteins were extracted from osteosarcoma cells with RIPA (Beyotime, China). Equal amounts of protein were denatured and separated by 12% SDS-PAGE. Then, the proteins were transferred to PVDF membranes. The PVDF membranes were then incubated with anti-CD44 or anti-β-actin (Abcam, U.K.) overnight at 4°C. After washing with TBST, the PVDF membranes were further probed with horseradish peroxidase-conjugated secondary antibodies (Stanta Cruz Biotechnology, U.S.A.). At last, intensity of blots was detected and quantified using an ECL detection system (Thermo Fisher, U.S.A.) at Quantity One Software (Bio-Rad, U.S.A.).

The article "GAPLINC is a predictor of poor prognosis and regulates cell migration and invasion in osteosarcoma" was published in 2018. Journal: Biosci Rep.

### Statistical analysis

All statistical analyses were performed with SPSS 17.0 statistical software. Data are presented as the mean ± S.D. The Wilcoxon Signed Rank test was applied for comparing the expression of lncRNA GAPLINC between OS tissue specimens and paired non-tumor tissue specimens. Two-tailed Student’s *t* test was used for comparisons of two independent groups. Chi-squared test was used to assess the association between GAPLINC expression and clinicopathological characteristics of osteosarcoma patients. Logrank test, univariate, and multivariate Cox regression were used in survival analysis. The *P* value <0.05 was considered as statistically significant.

## Results

### Levels of GAPLINC expression are increased in osteosarcoma tissues and cell lines

To investigate the status of GAPLINC expression in osteosarcoma tissues, we conducted RT-qPCR to detect GAPLINC expression in 40 pairs of osteosarcoma tissues and adjacent non-cancerous normal tissues. The result suggested that osteosarcoma tissues displayed higher levels of GAPLINC expression than adjacent non-cancerous normal tissues (*P*<0.001, Figure 1A). Then, we also measured GAPLINC expression in osteosarcoma cell lines (MG-63, HOS, SJSA-1, and Saos-2) and the human normal osteoblast cell line (hFOB1.19) through RT-qPCR, and found that GAPLINC expression was overexpressed in osteosarcoma cell lines (MG-63, HOS, SJSA-1, and Saos-2) compared with human normal osteoblast cell line (hFOB1.19) (*P*<0.001, Figure 1B).

**Figure 1:** Levels of GAPLINC expression are increased in osteosarcoma tissues and cell lines (**A**) Osteosarcoma tissues displayed higher levels of GAPLINC expression than adjacent non-cancerous normal tissues. (**B**) GAPLINC expression in osteosarcoma cell lines (MG-63, HOS, SJSA-1, and Saos-2) and the human normal osteoblast cell line (hFOB1.19).

### GAPLINC high-expression are correlated with clinical progression in osteosarcoma patients

To investigate the clinical significance of GAPLINC expression in osteosarcoma patients, levels of GAPLINC expression were detected in 126 clinical osteosarcoma tissue samples, and the relationship between GAPLINC expression and clinicopathological features was evaluated. The median expression level of GAPLINC in clinical osteosarcoma tissue samples was as the cutoff [17,18]. All samples were divided into two groups: high-expression of GAPLINC group and low-expression of GAPLINC group. As shown in Table 1, high-expression of GAPLINC was significantly associated with Enneking stage (*P*=0.026), distant metastasis (*P*=0.001), and histological grade (*P*=0.020). However, there was no statistical association of GAPLINC expression with age (*P*=0.857), gender (*P*=0.709), tumor size (*P*=0.201), and tumor site (*P*=0.364).

The article "GAPLINC is a predictor of poor prognosis and regulates cell migration and invasion in osteosarcoma" was published in 2018. Journal: Biosci Rep.

**Table 1:** Association between GAPLINC expression and clinicopathological characteristics in osteosarcoma cases

Characteristics	*n*	High-expression (%)	Low-expression (%)	*P*
**Age (y)**				
≤18	53	27 (50.9)	26 (49.1)	0.857
>18	73	36 (49.3)	37 (50.7)	
**Gender**				
Female	44	21 (47.7)	23 (52.3)	0.709
Male	82	42 (51.2)	40 (48.8)	
**Enneking stage**				
I-IIA	46	17 (37.0)	29 (63.0)	0.026
IIB-III	80	46 (57.5)	34 (42.5)	
**Tumor size**				
≤8 cm	77	35 (45.5)	42 (54.5)	0.201
>8 cm or discontinuous tumors	49	28 (57.1)	21 (42.9)	
**Distant metastasis**				
No	106	46 (43.4)	60 (56.6)	0.001
Yes	20	17 (85.0)	3 (15.0)	
**Histological grade**				
G1-G2	57	22 (38.6)	35 (61.4)	0.020
G3-G4	69	41 (59.4)	28 (40.6)	
**Tumor site**				
Femur/Tibia	102	49 (48.0)	53 (52.0)	0.364
Other	24	14 (58.3)	10 (41.7)	

### GAPLINC high-expression predicts poor clinical outcome in osteosarcoma patients

To investigate the prognostic value of GAPLINC expression in osteosarcoma patients, the association between GAPLINC expression and overall survival time was estimated. The result of logrank test showed that osteosarcoma patients with GAPLINC high-expression had poor overall survival compared with patients with GAPLINC low-expression (*P*<0.001, Figure 2). The risk factors of osteosarcoma patients were identified with univariate Cox regression analysis (Table 2). The results of univariate Cox regression analysis suggested that advanced Enneking stage (*P*<0.001), large tumor size (*P*=0.201), present distant metastasis (*P*<0.001), poor histological grade (*P*<0.001), and high-expression of GAPLINC (*P*<0.001) were poor prognostic factors in osteosarcoma patients. In order to assess the independent risk factors of osteosarcoma patients, we performed multivariate Cox regression analysis including Enneking stage, tumor size, distant metastasis, histological grade and present GAPLINC expression, and found that distant metastasis and GAPLINC expression were independent risk factors of osteosarcoma patients (*P*<0.001 and *P*=0.020, respectively).

**Figure 2:** GAPLINC high-expression predicts poor clinical outcome in osteosarcoma patients Kaplan–Meier survival curves revealed osteosarcoma patients with GAPLINC high-expression had poor overall survival compared with patients with GAPLINC low-expression.

**Table 2:** Univariate and multivariate Cox regression of prognostic factors for overall survival in osteosarcoma cases

Parameter	Univariate analysis			Multivariate analysis		
	HR	95% CI	*P*	HR	95% CI	*P*
**Age (y)**						
(≤18 compared with >18)	0.842	0.548–1.292	0.431			
**Gender**						
(Female compared with male)	1.401	0.886–2.217	0.150			
**Enneking stage**						
(I-IIA compared with IIB-III)	4.327	2.554–7.331	<0.001	2.407	1.040–5.572	0.040
**Tumor size**						
(≤8 cm compared with >8 cm or discontinuous tumors)	1.555	1.007–2.401	0.047	1.220	0.779–1.911	0.385
**Distant metastasis**						
(No compared with yes)	7.506	4.049–13.915	<0.001	3.977	2.065–7.658	<0.001
**Histological grade**						
(G1-G2 compared with G3-G4)	3.137	1.951–5.045	<0.001	1.299	0.634–2.662	0.474
**Tumor site**						
(Femur/Tibia compared with others)	1.406	0.834–2.372	0.201			
**GAPLINC expression**						
(Low compared with high)	2.984	1.909–4.663	<0.001	1.790	1.097–2.921	0.020

Abbreviations: 95% CI, 95% confidence interval; HR, hazard ratio.

The article "GAPLINC is a predictor of poor prognosis and regulates cell migration and invasion in osteosarcoma" was published in 2018. Journal: Biosci Rep.

### Knockdown of GAPLINC has no effect on osteosarcoma cell proliferation

To investigate the biological function of GAPLINC on osteosarcoma cell, loss-of-function experiments were conducted. Levels of GAPLINC expression in HOS and Saos-2 cells were relatively higher among four osteosarcoma cell lines (MG-63, HOS, SJSA-1, and Saos-2). Thus, HOS and Saos-2 cells were used for following loss-of-function experiments through transfection of siRNA-GAPLINC. Three siRNAs (si-1#, si-2#, and si-3#) were designed to down-regulate GAPLINC expression. The si-2# (siRNA-GAPLINC) was the most effective siRNA and was chosen for further experiments (Figure 3A). We performed CCK-8 assay to assess the effect of GAPLINC on cell proliferation, and found that knockdown of GAPLINC expression has no effect on cell proliferation in HOS and Saos-2 cells (*P*>0.05, Figure 3B).

**Figure 3:** Knockdown of GAPLINC has no effect on osteosarcoma cell proliferation (**A**) The transfection efficiencies of three siRNAs (si-1#, si-2#, and si-3#) were detected in HOS and Saos-2 cells. (**B**) Knockdown of GAPLINC expression has no effect on cell proliferation in HOS and Saos-2 cells.

### Knockdown of GAPLINC inhibits osteosarcoma cell migration, invasion, and CD44 expression

To investigate the effect of GAPLINC on osteosarcoma cell migration and invasion, cell migration and invasion assays were conducted in HOS and Saos-2 cells. The results of cell migration assay showed that the migration ability of osteosarcoma cell was obviously decreased when GAPLINC expression was decreased in HOS and Saos-2 cells (*P*<0.001, Figure 4A). Similarly, the invasion assay also suggested that knockdown of GAPLINC expression markedly suppressed the invasion ability of HOS and Saos-2 cells (*P*<0.001, Figure 4B).

**Figure 4:** Knockdown of GAPLINC inhibits osteosarcoma cell migration, invasion, and CD44 expression (**A**) Knockdown of GAPLINC expression markedly suppressed the migration ability of HOS and Saos-2 cells. (**B**) Knockdown of GAPLINC expression markedly suppressed the invasion ability of HOS and Saos-2 cells. (**C**) Knockdown of GAPLINC significantly reduced the protein level of CD44 in HOS and Saos-2 cells.

The article "GAPLINC is a predictor of poor prognosis and regulates cell migration and invasion in osteosarcoma" was published in 2018. Journal: Biosci Rep.

CD44 is a cell-surface glycoprotein that is overexpressed in most human tumors and modulates tumor cell metastasis via recruitment of CD44 to the cell surface [19]. Meanwhile, GAPLINC has been found to regulate CD44-dependent cell invasiveness [12]. Therefore, we investigated whether GAPLINC regulates osteosarcoma cell migration and invasion in a similar manner. We conducted Western blot to assess the effect of GAPLINC on CD44 protein expression, and found that knockdown of GAPLINC significantly reduced the protein level of CD44 in HOS and Saos-2 cells (Figure 4C).

## Discussion

GAPLINC is a novel lncRNA among aberrantly expressed lncRNAs in human gastric cancer specimens through the use of global microarray and *in situ* hybridization analyses [12]. Subsequently, Liu et al. [20] and Diao et al. [21] both confirmed that GAPLINC expression was up-regulated in gastric cancer tissues compared with normal gastric tissues. Meanwhile, Liu et al. [20] found that levels of GAPLINC expression were increased in poorly differentiated gastric adenocarcinoma tissues compared with highly differentiated gastric adenocarcinoma tissues. Moreover, several evidences showed that GAPLINC was also usually highly expressed in colorectal cancer tissues compared with adjacent normal tissues [13–15]. Besides, Zheng et al. [16] observed GAPLINC express was elevated in bladder cancer tissue compared with normal tissues through TCGA database, and the high levels of GAPLINC expression were confirmed in 80 pairs of bladder cancer tissues and adjacent normal tissues by RT-qPCR. However, the expression status of GAPLINC in osteosarcoma is still unknown. We performed RT-qPCR to measure the expression of GAPLINC in osteosarcoma clinical samples and cell lines, and found that levels of GAPLINC expression were increased in osteosarcoma clinical samples and cell lines compared with adjacent non-cancerous normal tissues and human normal osteoblast cell line, respectively. Then, we tried to explore the clinical significance of GAPLINC in osteosarcoma patients, and analyzed the relationship between GAPLINC expression and clinicopathological features. In our results, we observed that high-expression of GAPLINC was significantly associated with advanced Enneking stage, present distant metastasis, and poor histological grade. Similarly, Hu et al. [12] reported that GAPLINC high-expression was associated with large average tumor volume and severe invasion into lymph nodes in gastric cancer cases. In colorectal cancer patients, Yang et al. [14] found that high levels of GAPLINC expression were associated with large tumor size, advanced tumor stage (T classification), and advanced lymph node stage (N classification). Moreover, Zheng et al. [16] indicated that levels of GAPLINC expression were correlared with tumor stage in bladder cancer cases.

The article "GAPLINC is a predictor of poor prognosis and regulates cell migration and invasion in osteosarcoma" was published in 2018. Journal: Biosci Rep.

Recently, the prognostic value of GAPLINC expression has been suggested in gastric cancer [12,20], colorectal cancer [14], and bladder cancer [16]. Zheng et al. [16] demonstrated that bladder cancer patients in the high GAPLINC expression group had significantly shorter overall survival time than patients in the low GAPLINC expression group. Moreover, Hu et al. [12] and Liu et al. [20] congruously indicated that high-expression of GAPLINC was correlated with unfavorable prognosis in gastric cancer cases. Besides, Yang et al. [14] found that colorectal cancer patients with GAPLINC high-expression had a shorter overall survival than those with GAPLINC low-expression, and high-expression of GAPLINC served as an independent unfavorable prognostic factor for overall survival in colorectal cancer patients. Similarly, we also found osteosarcoma patients with GAPLINC high-expression had poor overall survival compared with patients with GAPLINC low-expression, and GAPLINC high-expression was an independent risk factor for osteosarcoma patients.

The biological function of GAPLINC in osteosarcoma cell remained unclear. Thus, we conducted loss-of-function experiments in osteosarcoma cell, and found that knockdown of GAPLINC inhibits osteosarcoma cell migration and invasion, but no effect on cell proliferation. In gastric cancer cell, GAPLINC has also been found to regulate CD44-dependent cell invasiveness [12,20]. CD44 is a cell-surface glycoprotein overexpressed in most human tumors and plays a key role in tumor cell adhesion and migration [19,22]. Therefore, we supposed that GAPLINC regulates osteosarcoma cell migration and invasion through modulating CD44 expression. In order to verify this hypothesis, we conducted Western blot to assess the effect of GAPLINC on CD44 protein expression, and found that knockdown of GAPLINC significantly reduced the protein level of CD44. Although GAPLINC has been found to positively regulate CD44 protein expression, the regulatory mechanism is still unknown. Thus, we will further explore the regulatory mechanism between GAPLINC and CD44 in regulating osteosarcoma cell migration and invasion in a future study.

In conclusion, GAPLINC expression is elevated in osteosarcoma tissues and cell lines, and correlated with the malignant status and prognosis. Knockdown of GAPLINC depressed osteosarcoma cell migration and invasion via inhibiting CD44 expression.

The article "GAPLINC is a predictor of poor prognosis and regulates cell migration and invasion in osteosarcoma" was published in 2018. Journal: Biosci Rep.

## Abbreviations

GAPLINC: gastric adenocarcinoma predictive long intergenic non-coding
lncRNA: long non-coding RNA
NC: negative control
RT-qPCR: real time polymerase chain reaction
TCGA: The Cancer Genome Atlas
